# Sleep Deprivation and Heart Rate Variability in Healthy Volunteers: Effects of REM and SWS Sleep Deprivation

**DOI:** 10.1155/2023/7121295

**Published:** 2023-07-11

**Authors:** YaHui Xu, BinBin Qu, FengJuan Liu, ZhiHua Gong, Yi Zhang, DeXiang Xu

**Affiliations:** ^1^Department of Respiratory and Critical Care Medicine, The Affiliated Central Hospital of Qingdao University, Qingdao, Shandong, China; ^2^Clinical Trial Research Center, The Affiliated Central Hospital of Qingdao University, Qingdao, Shandong, China; ^3^Electrocardiogram Department, The Affiliated Central Hospital of Qingdao University, Qingdao, Shandong, China; ^4^Department of Respiratory and Critical Care Medicine, Beijing China-Japan Friendship Hospital, China

## Abstract

**Objective:**

Using PSG-guided acute selective REM/SWS sleep deprivation in volunteers, this study examined the effects of sleep deprivation on the cardiovascular and autonomic nervous systems, as well as the relationship between cardiac neuromodulation homeostasis and cardiovascular disease.

**Methods:**

An experiment was conducted using 30 healthy volunteers (male : female = 1 : 1, aged 26.33 ± 4.5 years) divided into groups for sleep deprivation of SWS and REM sleep, and then, each group was crossed over for normal sleep (2 days) and repeated sleep deprivation (1 day, 3 times). During the study period, PSG and ELECTRO ECG monitoring were conducted, and five-minute frequency domain parameters and blood pressure values were measured before and after sleep deprivation.

**Results:**

Changes in VLF, LFnu, LF/HF, HF, and HFnu after SWS sleep deprivation were statistically significant (*P* < 0.05), but not LF (*P* = 0.063). Changes in VLF, LF, HF, LF/HF, LFnu, and HFnu after REM sleep deprivation were not statistically significant (*P* > 0.05).

**Conclusions:**

An increase in sympathetic nerve activity results from sleep deprivation and sudden awakening from SWS sleep is associated with a greater risk of cardiovascular disease.

## 1. Introduction

In addition to changes in awareness, sleep is characterized by a relatively inhibited sensory activity, decreased muscular activity, and inhibition of practically all voluntary muscles during fast eye movements, as well as decreased interaction with the surrounding environment [1]. It differs from wakefulness in that it is less responsive to stimuli, yet it is more reactive than comas or disturbing states of consciousness. As a result of sleep, the brain exhibits a different pattern of active activity [2]. A good night's sleep enhances the human body's energy and resistance, supports proper human growth and development, and ensures that the human body receives sufficient rest. It is impossible to overestimate the importance of sleep in maintaining mental activity and protecting mental health [3, 4]. Getting enough sleep and maintaining good sleep quality can help maintain a normal metabolism and reduce the occurrence and mortality of certain diseases. It has become increasingly evident that sleep deprivation (SD) is a serious public health issue [5]. Aging, lifestyle, time stress, shift work, insomnia, and sleep disorders are all factors that contribute to insufficient sleep, microawakening, and fragmented sleep [5, 6]. In addition to cardiovascular disease, obesity, and diabetes, SD can also increase the risk of depression. Clinical trials have shown that SD can weaken the autonomic nervous system and change the stability of the cardiovascular system [7]. Heart rate changes and the maintenance of cardiac sinus rhythm are primarily regulated by sympathetic and parasympathetic nerves. In terms of cardiac autonomic nerve regulation analysis, heart rate variability (HRV) is the best noninvasive monitoring method [8]. Studies examining cardiovascular neuromodulation during sleep have been widely evaluated using 5-minute frequency domain analysis [9]. According to the literature, the sympathetic nervous system is enhanced after acute sleep deprivation, and the vagal nerve is decreased after acute sleep deprivation [5]. However, there is a significant difference between the activity of sympathetic and parasympathetic nerves during different sleep stages, and the effects of sleep deprivation on the autonomic nervous system in different sleep stages have not been reported. By analyzing heart rate variability 5 minutes before and after selective sleep deprivation (frequency domain analysis), this study investigated the relationship between acute selective sleep deprivation HRV and cardiovascular disease.

## 2. Methods

### 2.1. Samples and Standards

This study has been approved by the Medical Ethics Committee of Qingdao Central Hospital (Ethics Review Approval No. Ky-p201807501), and the clinical trial has been registered online (registration number ChiCTR1900020622). Prior to explaining the purpose and procedure of the study to the healthy subjects, healthy volunteers were recruited, and the study was conducted between February 2019 and December 2020. During the clinical screening process, patients undergo a detailed history and physical examination in addition to basic examinations (heart function, blood pressure, electrocardiogram, lung function, etc.) and evaluation questionnaires.

### 2.2. Criteria for Inclusion and Exclusion

Criteria for inclusion are as follows: between 20 and 39 years of age, one week of stable sleep prior to the experiment, no shift work during the preceding three months, and one week of stable daily activities and work prior to the experiment. Criteria for exclusion are as follows: a BMI of more than 30 kg/m^2^, acute or chronic cardiopulmonary diseases, smoking more than ten cigarettes per day, alcoholism, consuming more than 100 g of alcohol per week, recent negative life events, physical and neurological examinations that are abnormal, mothers who are pregnant or nursing, and any sleep-related breathing disorder. The study protocols for the examinations were conducted in accordance with the Helsinki Declaration (2000), and the participants were compensated monetarily upon completion of the tests.

### 2.3. Sleep Intervention

30 volunteers (male: female ratio of 1 : 1, mean age of 26.3 ± 4.5 years) who met the inclusion and exclusion criteria were randomly assigned to either the REM sleep deprivation or SWS sleep deprivation group. Prior to the trial, all subjects were instructed to maintain a regular sleep schedule between 10 : 00 p.m. and 7 : 00 a.m. Trials were conducted for three days: normal sleep on day one (excluding the effects of first night sleep and screening for exclusion criteria during sleep), selective sleep deprivation on day two, and normal sleep after sleep deprivation on day three. In the event of sleep restriction and normal sleep, PSG monitoring was performed in order to determine sleep stages, and a dynamic electrocardiogram was worn in order to evaluate autonomic nervous system indicators. Monitoring took place from 21 : 00 to 7 : 00 the following morning. During the night of sleep deprivation, volunteers woke up after entering SWS sleep or REM sleep. Sensei's methods were to turn on the light, and by playing a specific decibel of ringtones and vibration signals, wake up the loser for three minutes of artificial intervention, let it stay awake for five minutes, and then, turn off the light into the next round of sleep. Three times a night, they were deprived of sleep. Blood pressure monitoring: during sleep and after waking, the blood pressure is monitored in terms of systolic and diastolic values.

### 2.4. Data Collection

Data from polysomnography (PSG) was recorded simultaneously in order to assess sleep phases. A dynamic ECG recorder (CT-086, CT-082, and CT-083s) was developed by Hangzhou Baihui Medical Equipment Co., Ltd. The data was analyzed using the company's most recent software (V1.0.0), and the recording period was from 21 : 00 to 07 : 00 in the evening. An analysis of the frequency domain of the dynamic ECG was performed in order to determine the HRV. During and after sleep deprivation, continuous 5-minute HRV frequency domain data was analyzed without interruption. In addition to the VLF (very low frequency), LF (low frequency), HF (high frequency), and LF/HF (low frequency/high frequency) ratios, the LFnu (standardized low-frequency component) and HFnu (standardized high-frequency component) represent sympathetic tone. HF is a marker of cardiac vagal tone, and the LF/HF ratio is a more sensitive indicator of sympathetic nerves.

### 2.5. Statistical Analysis

For the statistical analysis, SPSS24.0 statistical software was used. In this study, the measurement data of normal distributions were expressed as *X* ± *S*. A paired *T*-test was used to compare quantitative data with a normal distribution before and after treatment, and *P* < 0.05 was considered statistically significant.

## 3. Results

### 3.1. Analysis of Patient Data Using Statistical Methods

The study recruited 30 qualified participants from a pool of fifty healthy participants. In the SWS sleep deprivation group, one individual was eliminated from the study due to a lack of slow-wave sleep on the night of sleep deprivation, resulting in a total of 29 subjects being included in the analysis. As shown in Table 1, healthy individuals have the following baseline characteristics.

### 3.2. An Analysis of the HRV Frequency Domain for Five Minutes

As compared with before deprivation, VLF, LFnu, and LF/HF increased after sleep deprivation, whereas HF and HFnu decreased, and the difference was statistically significant (*P* < 0.05). There was a significant difference between the LF/HF before SWS deprivation and the LF/HF before REM deprivation. In contrast, the LF/HF after SWS deprivation was significantly higher than the LF/HF after REM deprivation, as shown in Table 2. Table 2 shows that there was no statistical significance between before and after REM sleep deprivation in VLF, LF, HF, LF/HF, LFnu, or HFnu in the REM sleep deprivation group (*P* > 0.05).

Heart rate variability is measured through HRV (heart rate variability), VLF (extremely low frequency), LF (low frequency), HF (high frequency), LF/HF (low-frequency to high-frequency ratio), LFnu (normalized low-frequency component), and HFnu (normalized high-frequency component).

### 3.3. The Results of Changes in Blood Pressure

A significant difference (*P* < 0.05) was found between the diastolic blood pressure after waking after SWS and REM sleep deprivation, as shown in Table 3.

## 4. Discussion

An adult experiences four to six cycles of REM and non-REM sleep during the night, and increased dopamine (DA) secretion in the basolateral amygdala (BLA) terminates SWS sleep and initiates REM sleep [9]. The sympathetic nervous system is primarily responsible for regulating REM sleep, and sympathetic activity may result in dramatic fluctuations in cardiopulmonary function [10, 11]. Consequently, sleep deprivation has been linked to cardiovascular disease in epidemiological studies, but the extent of the association is unclear [12].

There have been several studies suggesting that sleep deprivation may increase blood pressure, regardless of whether the deprivation is complete or partial [13, 14]. Five healthy adults were subjected to partial sleep deprivation (4.2 hours of nighttime sleep) by Meier-Ewert et al. [15]. It was found that the systolic blood pressure and heart rate increased as well as the high-sensitivity C-reactive protein (CRP) level during sleep deprivation. There is evidence to suggest that sleep deprivation may activate inflammatory processes and therefore result in an increase in cardiovascular disease incidence.

According to our findings, SWS sleep deprivation decreases vagal innervation activity and increases sympathetic activity, such as decreased HF, increased LF to HF ratio, and decreased LFNU and HFNU, reflecting sleep deprivation's subtle effects on cardiovascular health that are difficult to capture through clinical assessments. The HRV-related indicators (VLF, LF, HF, LF/HF, LFnu, and HFnu) did not differ statistically significantly after REM sleep deprivation, which may be explained by the dominance of sympathetic activity during REM sleep deprivation. A study by Scholz et al. [16] found that LF/HF began to increase even 15 minutes before REM sleep, suggesting that the risk of cardiovascular disease may be associated with REM sleep, which may also explain the higher rate of cardiovascular events in the morning [17]. A typical eight-hour sleep cycle includes 90 to 120 minutes of REM sleep, which means that there is a higher risk of sudden death, up to 1.2 times that of awakened sleep [18]. It is assumed that sympathetic innervation is enhanced during REM sleep than during SWS sleep due to the body's physiological waking activity, since LF/HF values decrease after SWS sleep deprivation but remain higher than those after REM sleep deprivation. According to current theories, the body's physiological regulation of waking activity enables it to avoid a surge in sympathetic activity levels during sudden awakening as a result of increased sympathetic innervation during REM sleep compared to SWS sleep. Sudden awakening from slow-wave sleep causes greater fluctuations in autonomic activity, and an increased cardiovascular risk is associated with sudden awakening from slow-wave sleep in vulnerable individuals. It is consistent with the experimental results of Goff et al. [19] who found that waking from slow-wave sleep was associated with more dramatic fluctuations in blood pressure in the morning than waking from rapid eye movement sleep. Consequently, a sudden change in autonomic nervous system innervation during transitions between deep sleep and light sleep or awakening may result in adverse cardiac events in patients with severe impaired autonomic nervous system function [20].

Pure diastolic hypertension has been reported, especially in the early stages of sleep-disordered breathing, as a specific pattern of hypertension associated with the disease [21], and DBP may be an early indicator of cardiovascular outcomes in OSA patients. Elevated DBP is generally associated with increased peripheral resistance, which is primarily determined by the arterial vessels, whereas elevated SBP is primarily determined by the large and medium vessels [22, 23]. In the absence of elevated SBP, DBP increases suggest that repeated sleep deprivation has a greater impact on the peripheral vasculature than the large to medium vessels. In this study, blood pressure studies after selective sleep deprivation indicated that following repeated deprivation of SWS and REM sleep for three times, postwake DBP was higher than prewake DBP, while changes in SBP were not statistically significant, which suggests that peripheral resistance and fluctuation in blood pressure are caused by sympathetic activation [24]. Nevertheless, changes in sympathetic nerve activity are not always accompanied by changes in blood pressure, and more research is necessary to determine the exact mechanisms behind these changes.

Several health risks are associated with sleep deprivation, including cardiovascular, respiratory, neurological, gastrointestinal, immune, cutaneous, endocrine, and reproductive health [25]. As the number of indicators for analysis in our study was limited, we intend to expand the cohort to include more indicators in our next study in order to obtain clinical data.

## 5. Conclusions

As a result of REM/SWS sleep deprivation, diastolic blood pressure increased. Various HRV parameters are associated with different sleep stages after sleep deprivation. For example, the REM period is not significantly affected by sleep-related parameters of HRV after sleep deprivation of the SWS period. People with a healthy autonomic nervous system are better able to tolerate this fluctuation, whereas people with a vulnerable autonomic nervous system are at a higher risk of cardiovascular events as a result of slow-wave sleep. Due to the increased sympathetic activity of REM sleep compared to NREM sleep, the impact of REM sleep on patients at high risk of cardiovascular disease cannot be overlooked. Therefore, cardiac monitoring and advance intervention are important in high-risk patients during different sleep periods at night in order to reduce the occurrence of adverse events. In addition, we will further investigate the changes in hemodynamics and related factors during different sleep periods and the specific mechanisms of cardiovascular events during different sleep periods.

## Figures and Tables

**Table 1:** Baseline characteristics of healthy volunteers.

Factor	Mean ($\bar{X}\pm S$)
Age (y)	26.27 ± 4.479
Height (cm)	168.93 ± 7.803
Weight (kg)	65.53 ± 13.568
BMI (kg/m^2^)	22.76 ± 3.283
HR (bpm)	72.53 ± 8.561
SBP (mmHg)	114.80 ± 12.344
DBP (mmHg)	70.73 ± 9.381

**Table 2:** Analyses of 5-minute HRV frequency domains before and after selective sleep deprivation in volunteers ($\bar{X}\pm S$).

Project	REM deprivation (before)	REM deprivation (after)	*P*	SWS deprivation (before)	SWS deprivation (after)	*P*
VLF	2925 ± 2724	3524 ± 2425	0.403	808 ± 665	2299 ± 1745	0.003
LF	974 ± 612	1005 ± 603	0.867	608 ± 433	1048 ± 854	0.063
HF	1273 ± 670	916 ± 676	0.387	1169 ± 571	548 ± 214	0.001
LF/HF	1.42 ± 1.01	1.65 ± 2.09	0.665	0.58 ± 0.49	2.05 ± 1.43	0.005
LFNU	52.50 ± 16.70	52.87 ± 14.92	0.94	33.20 ± 3.61	59.63 ± 19.23	0.002
HFNU	47.50 ± 16.70	46.93 ± 14.85	0.909	66.80 ± 13.50	40.37 ± 19.23	0.002

**Table 3:** The effects of selective sleep deprivation on blood pressure in 30 healthy volunteers ($\bar{X}\pm S$).

Project	REM deprivation		SWS deprivation	
	SBP (mmHg)	DBP (mmHg)	SBP (mmHg)	DBP (mmHg)
BP before sleeping	106.07 ± 11.32	62.13 ± 5.25	105.00 ± 11.09	62.40 ± 5.22
BP after waking	108.87 ± 11.29	67.80 ± 8.03	108.67 ± 11.70	66.27 ± 1.71
*P*	0.134	0.038	0.117	0.019

## Data Availability

Datasets used in the current study may be obtained from the corresponding author upon request.
